The article "Clinical Study of Airway Stent Implantation in the Treatment of Patients with Malignant Central Airway Obstruction" was published in 2022. Journal: Evid Based Complement Alternat Med.

# Clinical Study of Airway Stent Implantation in the Treatment of Patients with Malignant Central Airway Obstruction

**DOI:** 10.1155/2022/6933793

**Published:** 2022-08-10

**Authors:** Yuanyuan Xing, Xuedong Lv, Daxiong Zeng, Junhong Jiang

**Affiliations:** ^1^Department of Pulmonary and Critical Care Medicine, The First Affiliated Hospital of Soochow University, Suzhou, Jiangsu 215000, China; ^2^Department of Emergency Medicine, The Second Affiliated Hospital of Nantong University, Nantong, Jiangsu 226001, China; ^3^Department of Pulmonary and Critical Care Medicine, Dushu Lake Hospital Affiliated to Soochow University, Suzhou, Jiangsu 215000, China

## Abstract

**Background:**

Airway stenting is a therapeutic option for malignant central airway obstructions (MCAO), including both intraluminal and extraluminal obstructions. The objective of this study is to investigate the clinical features and results of long-term improved prognosis for MCAO patients after airway stent implantation.

**Methods:**

Ninety-eight MCAO patients who underwent stent placement in our hospital from January 2013 to April 2020 were included in this study. The data included baseline data, clinical characteristics, laboratory test data, stent implantation data, and treatment as well as survival after stent implantation. The survival rates among individuals were compared via log-rank tests. Potential prognostic factors were identified using multivariate cox hazard regression models.

**Results:**

A retrospective analysis of these patients was generated. MCAO was mainly caused by lung cancer (53/98, 54.08%), esophageal cancer (22/98, 22.45%), and thyroid cancer (3/98, 3.06%). The median survival time of participants was 5.5 months. Univariate analysis indicated that the survival rate was related to primary disease, ECOG PS score, stent site, hemoglobin (Hb), albumin (ALB), and serum lactate dehydrogenase (LDH) (*P* < 0.05). The cox risk regression model showed that the survival rate was significantly influenced by ECOG PS score (OR = 3.468, 95%CI = 1.426–8.432, *P* = 0.006) and stent site (OR = 1.544, 95%CI = 1.057–2.255, *P* = 0.025).

**Conclusions:**

Compared with the site of stent placement, the ECOG PS score is the primary factor in the survival rate of MCAO patients after airway stenting.

## 1. Introduction

For patients with thoracic malignant tumors, malignant central airway obstruction (MCAO) was mainly caused by intraluminal tumor growth or external tumor compression [1]. Airway stents maintain airway patency by interrupting tumor expansion or preventing malignant tumor compression, which is a palliative treatment for MCAO to improve symptoms, quality of life, or lung function [2, 3]. Stent placement can improve MCAO for patients with malignant tumors. It is a challenge to place an artificial stent in the airway since serious risks exist in stent implantation, including bleeding, intraoperative airway obstruction, and dislocation or migration from the desired site [4]. Therefore, the indications for stent placement in thoracic malignancies should decide on risks and benefits. Although airway stent placement has been mainly used as palliative treatment, the prognostic benefit of stent placement is still controversial [5]. At present, many studies on airway stents have focused on palliative care, lung function, risks, and complications after stent placement, while factors of survival remain confused [6]. For instance, Nagano reported that only good performance status contributed to survival after airway stent placement, of which only 21 patients were analyzed [7]. Herein, factors to determine the clinical features and improve the long-term prognosis for MCAO patients treated with airway stent implantation were performed in this paper.

The article "Clinical Study of Airway Stent Implantation in the Treatment of Patients with Malignant Central Airway Obstruction" was published in 2022. Journal: Evid Based Complement Alternat Med.

Malignant central airway stenosis (MCAS) refers to the primary malignancy of the trachea, the left and right main bronchus and the right middle bronchus, or the malignant external pressure of the peritracheal tissues and organs, as well as the airway stenosis and obstruction caused by the metastasis of the peritracheal tissues and organs or tumors in other parts. Obstruction of the airway by tumor tissue will lead to difficulty in ventilation, which is manifested as chest tightness and shortness of breath. In severe cases, it can lead to respiratory failure and even endanger the patient's life. It is a common emergency in clinic. Such patients have severe symptoms, high treatment risk, and poor prognosis, and the key to clinical treatment is the rapid removal of airway obstruction.

There are many malignancies that threaten human health. Lung cancer is one of the most common types. According to statistics, in recent years, lung cancer has the fastest incidence and death rates and has become one of the most harmful malignant tumors to human life and health. In patients with lung cancer, about 30% of patients will progress to develop atmospheric airway stenosis.

Chemotherapy and extracorporeal radiotherapy are an option for cancer patients who cannot undergo a surgery. However, they are slow to start and are not suitable for patients with respiratory distress and even asphyxia. With the continuous development of the airway endoscopic technology, many intraluminal interventional techniques have gradually emerged, such as the internal airway stent implantation, particle implantation, laser, high-frequency electric knife, argon knife, freezing, photodynamic therapy, and other technical means.

The article "Clinical Study of Airway Stent Implantation in the Treatment of Patients with Malignant Central Airway Obstruction" was published in 2022. Journal: Evid Based Complement Alternat Med.

## 2. Methods

### 2.1. Ethical Statement

The study was conducted in accordance with the Declaration of Helsinki (as revised in 2000), which was approved by the First Affiliated Hospital of Soochow University (No. 2021[336]). Informed consent was obtained from all individual participants involved in the study.

### 2.2. Study Population and Data Collection

All participants underwent stent placement for MCAO in our hospital from January 2013 to April 2020. Clinical data and follow-up information were obtained from medical records or telephone interviews with family members of patients. The criteria for recruiting patients in this study were as follows: (i) MCAO was determined using bronchoscopy or chest computed tomography (CT); the symptom of cross-sectional area of the lumen decreased by more than 50%, or obvious dyspnea could be observed; (ii) patients received airway stents placement surgery. Patients with incomplete clinical data would be excluded.

The data collected from each patient included baseline data (gender, age, body mass index (BMI), smoking history, and basic comorbidities), clinical characteristics (causes, prestent ECOG PS score), laboratory test data (hemoglobin (Hb), albumin (ALB), and serum lactate dehydrogenase (LDH)), stent placement (location and complications), and treatment and survival rate after stent placement. The evaluation of ECOG PS score before stent implantation was referred to the previous method [8].

### 2.3. Airway Stent Implantation

All patients underwent chest CT and soft bronchoscopy to assess the severity of MCAO before stent placement. For patients with local anesthesia or general anesthesia, the stent (straight, L-shaped, or Y-shaped metal airway stent) was delivered to the quasi-lesion site under bronchoscope or X-ray guidance. The airway with significant obstruction could be treated with airway intervention, such as balloon dilation, before stent placement. Due to the technical and material limitations, the stents used in this study were all metal airway stents obtained from Nanwei Medical Technology Co., Ltd.

### 2.4. Postoperative Monitoring

Routine bronchoscopy was performed one week after stent placement to check the status of the stent and refractory secretions. MCAO recurrence would be caused by tumors, granulation tissue formation, or refractory secretions after the initial stent implantation. To maintain airway patency, bronchoscopy intervention would be performed, including argon plasma coagulation (APC), laser, and stent replacement, cryotherapy.

### 2.5. Statistical Analysis

SPSS 22.0 was used for statistical analysis. Continuous variables were presented as mean ± standard deviation, and categorical variables were frequency (%). The survival time began from the placement of stent to the death of patient or the last follow-up of the living patient, and the last follow-up for this study was in November 2020. The overall survival rate was represented by the Kaplan-Meier curve. The log-rank test was used to analyze the survival rate between each subgroup of potential prognostic factors. Later, the factors (*P* < 0.05) that were based on the log-rank analysis and probably affected the prognosis were analyzed via the multivariate Cox risk regression model based on the forward stepwise regression with maximum likelihood estimation. The results of the potential predictors were presented with hazard ratios (OR) and 95% confidence interval (CI). The level of statistical significance was set at two-tailed *P* < 0.05.

The article "Clinical Study of Airway Stent Implantation in the Treatment of Patients with Malignant Central Airway Obstruction" was published in 2022. Journal: Evid Based Complement Alternat Med.

Chronic infectious diseases caused by tuberculosis bacteria are called *tuberculosis*. Respiratory transmission is the main mode of transmission of this disease, and young people are more prone to TB. *Tuberculosis bacillus* can invade any organ in the human body or the whole body. It often invades the lung. Conjunctival disease refers to tuberculosis occurring in the trachea, bronchial mucosa, submucosa, smooth muscle, cartilage, and adventitia, which is called trachea and bronchial tuberculosis (tracheobronchial tuberculosis, TBTB).

Airway stenosis has traditionally been treated by surgery. Surgical resection of tracheal stenosis and suture of broken ends are the classic methods to treat tracheal stenosis. Although the surgical treatment can solve airway stenosis quickly and effectively, it also has the disadvantages of large trauma, many complications, and high cost, which some patients do not easily accept. With the progress of medicine, especially the rapid development of interventional technology, bronchial interventional treatment of airway stenosis has attracted more and more attention because it can make up for the shortcomings of traditional surgical treatment.

## 3. Results

### 3.1. Assessment of Clinical Data and Survival Rate

Ninety-eight consecutive patients aged 33 to 83 years were included, with an average age of 65.07 ± 8.89 years, and the ratio of male to female was 74 : 24. The body mass index ranged from 15.94 to 32.03 kg/m^2^, the mean of which was 21.72 kg/m^2^. Thirty-five patients (35.71%) had a history of smoking. In this study, MCAO was mainly caused by lung cancer (53/98, 54.08%), esophageal cancer (22/98, 22.45%), and thyroid cancer (3/98, 3.06%), with the basic comorbidities of hypertension (46/98, 46.94%), diabetes (11/98, 11.22%), coronary heart disease (4/98, 4.08%), chronic lung disease (4/98, 4.08%), *tuberculosis* (2/98, 2.04%), prostate hyperplasia (2/98, 2.04%), and other diseases (9/98, 9.18%). One or two stents were implanted in each patient, bringing the total of metal stents to 10^8^. ECOG PS score indicated that 80 cases (81.63%) had a score of 0–2, while 18.37% had a score of 3–4.

The article "Clinical Study of Airway Stent Implantation in the Treatment of Patients with Malignant Central Airway Obstruction" was published in 2022. Journal: Evid Based Complement Alternat Med.

The characteristics of airway stent placement in MCAO were summarized to further analyze the factors of survival (Table 1). Most stent placements were performed under local anesthesia (73.47%). The main stent sites were the trachea (46/98, 46.94%), the left main bronchus (19/98, 19.39%) and the right main bronchus (21/98, 21.43%). Complications after stent placement included neoplasms (36/98, 36.73%), sputum (30/98, 30.61%), mucus secretions (28/98, 28.57%), granulation tissue formation (21/98, 21.43%), necrosis (14/98, 14.29%), tumor endo growth (8/98, 7.14%), fistula (6/98, 6.12%), and stent displacement (3/98, 3.06%). After stent placement, there were 22 cases (22.45%) without any treatment, 21 cases (21.43%) were treated with chemotherapy, 14 cases (14.29%) for radiotherapy, 31 cases (31.63%) received radiotherapy and chemotherapy, and seven cases (7.14%) were given only supportive treatment.

It all depends mainly on the nature and scope of the lesion. It is closely related to the site and degree of lumen stenosis. At the beginning of the disease, when the scope of lesions is relatively small, the patient does not have any clinical symptoms. With the development of the disease, when the scope of exudative lesions expand, or caseous necrosis develops, it is manifested as hyperemia and edema of the tissue, infiltration of neutrophils, lymphocytes and monocytes, exudation of fibrin, and a small number of epithelioid cells and multinucleated giant cells. Acid fast staining can detect *Mycobacterium tuberculosis*.

Clinically, the chest *X* tablet is the most basic examination except for lung diseases. The *X* tablets in patients with bronchial *tuberculosis* are mostly complicated with pulmonary *tuberculosis* lesions, which can appear as exudative lesions, caseous lesions, tuberculous nodules, or nodular granuloma. Most of the bronchial *tuberculosis X* tablets cannot show direct signs of airway stenosis and mostly show indirect symptoms, such as localized pulmonary atelectasis and obstructive pneumonia.

Ninety-three patients died, and five patients were still alive till the end of the study. The median survival time was 5.5 months. The survival rates at 1, 3, 6, 9, 12, 24, 36, and 60 months were 79.73%, 63.51%, 43.24%, 37.84%, 29.73%, 15.17%, 7.59%, and 3.79%, respectively. The overall survival curve indicated that the cumulative survival rate decreased with time (Figure 1).

The article "Clinical Study of Airway Stent Implantation in the Treatment of Patients with Malignant Central Airway Obstruction" was published in 2022. Journal: Evid Based Complement Alternat Med.

### 3.2. Univariate Log-Rank Test Analysis of Survival Rate

Univariate analysis of potential prognostic factors in 98 patients showed that the survival rate of participants was related to the primary disease, ECOG PS score, the site of stent, Hb, ALB, and LDH (*P* < 0.05) (Table 2). The survival curve estimated by Kaplan-Meier was shown in Figure 2.

### 3.3. Multivariate Cox Regression Analysis of Survival Rate

Select factors related to survival of MCAO patients after airway stent placement by univariate analysis (*P* < 0.05) and other factors mentioned in previous studies or considered to have an impact on the prognosis are mentioned in Table 3]. Variable cox risk regression model was used for further analysis. Multivariate analysis showed that ECOG PS score (OR = 3.468, 95%CI = 1.426–8.432, *P*=0.006) and stent site (OR = 1.544, 95%CI = 1.057–2.255, *P*=0.025) were significantly related to the survival rate (Table 4).

## 4. Discussion

MCAO patients were on the low edge of survival rate, and their the median survival time without any treatment was only one to two months [9, 10]. Bronchoscopy interventional techniques have been developed to reduce the mortality rate of MCAO and prolong the lives of patients by providing more opportunities for further antitumor therapy [11]. The studies on airway stents in the treatment of MCAO are all retrospective because of the difficulty to conduct prospective and large-scale studies as well as the small base of patients.

Chest CT, especially high-resolution CT (high resolution CT, HRCT), can significantly improve the disease diagnosis. The HRCT imaging of bronchial *tuberculosis* usually shows the thickening of the bronchial tube wall, which then leads to lumen stenosis, atelectasis, and obstructive pneumonia. The patient undergoes a tracheal tomography in the anterior and posterior, lateral, and oblique positions, which can show the site and extent of the stenosis and help clinicians understand the length and morphology of the bronchus. HRCT can also show the number and range of the affected bronchi and whether the lymph nodes are involved and complications.

Husain reported that seven of 46 MCAO patients were alive after treatment with Ultraflex metal stents, with a median survival time of 128 days, ranging from 3 to 1859 days [12]. Saji conducted a retrospective study that included 65 patients with advanced lung cancer in MCAO, in which a survival rate of 25.2% in one year and a median survival rate of 6.2 months were obtained [13]. Inchingolo presented a retrospective study of 140 patients with malignant tumors, including 107 non-small cell carcinomas, nine small cell carcinomas, nine lymphomas, eight esophageal cancers, and seven intrabronchial metastases, while the 1-year survival rate was 15% and the median survival time after stent placement was 3.4 months [14]. In this study, the common diseases that mainly resulted in MCAO included lung cancer (54.08%), esophageal cancer (22.45%), and thyroid cancer (3.06%). The median survival time of patients after stent implantation was 5.5 months, which is close to 4.7 months reported by Guibert [15].

The article "Clinical Study of Airway Stent Implantation in the Treatment of Patients with Malignant Central Airway Obstruction" was published in 2022. Journal: Evid Based Complement Alternat Med.

The diagnosis of bronchial *tuberculosis* relies on the comprehensive analysis of epidemiology, medical history, clinical manifestations, physical signs, and related auxiliary examinations (such as sputum search for *Mycobacterium tuberculosis*, chest imaging, PPD, T cell spot experiment, and bronchoscopy). Because the clinical manifestations of bronchial *tuberculosis* patients often lack specificity, and the imaging examination has its limitations, the current diagnosis of bronchial *tuberculosis* mainly depend on bronchoscopy, bacteriological, or pathological evidence.

Due to the slow onset of bronchial *tuberculosis*, diverse manifestations, and lack of specificity, grassroots doctors have limited diagnosis and treatment levels, so patients are prone to misdiagnosis. If bronchial *tuberculosis* is not adopted by timely and standardized diagnosis and treatment, once the scar stenosis or tube wall softening occurs, lung ventilation dysfunction can occur. In severe cases, repeated lung infection, lung atresia, and lung damage caused by obstructive pneumonia may even occur, which seriously affects the quality of life of patients.

Bronchoscopy interventional techniques have been seen as one of the positive prognostic factors of MCAO patients. In addition, independent prognostic factors for MCAO patients with interventional bronchoscopy have been reported, such as the etiology, ASA score, obstruction site, external or mixed lesions, preoperative adjuvant therapy, and preoperative ECOG PS score as well as treatment [16, 17]. Compared with the previously mentioned studies, this study focused on MCAO patients undergoing stent implantation and excluded the influence of other interventions. Furthermore, the preoperative ECOG PS score and the stent placement site also influenced the independent prognosis for MCAO patients after airway stent placement.

Some patients with bronchial *tuberculosis* have chest tightness, urgent breath, or dyspnea when diagnosed, and only oral antituberculosis drugs are often effective slowly and take longer than *tuberculosis* treatment, which is easy to delay the disease and increase the sequelae. In order to prevent the formation of airway stenosis, shorten the course of treatment, and significantly improve the quality of life of patients, the bronchoscope airway intervention technology is usually continued to be used for local treatment on the basis of systemic chemotherapy.

The article "Clinical Study of Airway Stent Implantation in the Treatment of Patients with Malignant Central Airway Obstruction" was published in 2022. Journal: Evid Based Complement Alternat Med.

The indications are suitable for patients with ulcerative necrotic and granulation proliferative bronchial *tuberculosis* airway stenosis. Some of the disadvantages of the current microwave treatment operation equipment, which limit its use in the previously mentioned cases, are as follows: microwave radiation range is small, larger lesions need repeated operations, it increases the workload of medical staff and causes operation inconvenience, and it can easily cause tube wall perforation, tracheoesophageal fistula, or complications such as cold light source burns.

The ECOG PS score was not only an indicator to determine whether cancer patients should receive chemotherapy but also a prognostic factor for cancer patients [18]. Similar to the study reported by Ong, this study showed that patients with a high ECOG PS score [3, 4] had a worse prognosis than patients with a low ECOG PS score [0–2] (the mean survival time was 3.85 months and 12.35 months, resp., *P*=0.004), indicating that patients with good PS might survive from stent implantation to prolong survival and improve oxygenation [19]. Stent placement has been proven to prevent acute asphyxia, reduce the patient's fear of sudden death, and provide patients with enough time to receive additional treatments, such as chemotherapy, radiotherapy, and palliative care [20]. Indications of airway stent implantation should be determined carefully for patients with poor PS. Although stent implantation could alleviate severe dyspnea symptoms, patients with high PS scores might have fewer opportunities to receive antitumor therapy, and survival time after surgery was probably still short.

Mohan reported that the location of the lesion not only determined the type (straight, *L* or *Y*) and length of the airway stent but also affected the independent predictors of survival in MCAO patients. This study showed a worse prognosis for patients with both trachea and main bronchus than those who were only placed one stent in the trachea (average survival time was 15.23 months and 1.25 months, resp.), which indicates that compound MCAO (striction of both trachea and main bronchus) was more serious than simple MCAO (striction of trachea or main bronchus only).

Research by Wang reported that the antitumor therapy prolonged the survival time of MCAO patients with the intervention of airway stent implantation (*P* < 0.001), while the effect of different antitumor therapies on the prognosis for these MCAO patients after bronchoscopy intervention was not presented [21]. Our study supplemented this data and showed that the average survival time of the radiotherapy and radiochemotherapy groups after stent placement was 15.33 and 11.61 months, respectively, which exceeded the 5.00 months of the only supportive treatment group. However, the average survival period of the chemotherapy group after stent placement was close to that of the supportive treatment group, probably since most cases were in the terminal stage, and nearly half of the patients received chemotherapy before implanting the stent. As a local treatment method, radiotherapy is more effective than chemotherapy in controlling local airway stenosis. The results in our study indicated that a longer survival time existed in MCAO patients with radiotherapy rather than chemotherapy after stent placement, which meant that the radiotherapy counted for these patients as a local treatment to maintain airway patency, especially to those who received chemotherapy before or after stent placement.

The article "Clinical Study of Airway Stent Implantation in the Treatment of Patients with Malignant Central Airway Obstruction" was published in 2022. Journal: Evid Based Complement Alternat Med.

Certain limitations in this study were as follows. (i) This was a single-center, retrospective study, and more multicenter and prospective studies are needed. (ii) Different tumors respond differently to radiotherapy and chemotherapy, which might result in the various data obtained from different participants. Despite these limitations, we obtained the important finding that the ECOG PS score before stent placement and the site of stent placement affected the survival rate of MCAO patients. Therefore, stent implantation was more beneficial to patients with lower ECOG PS scores before stent implantation and simple MCAO patients.

## 5. Conclusion

This study included 98 MCAO patients after stent placement to investigate the clinical features and results of long-term improved prognosis. The results from this study demonstrate a regular trend regarding the baseline characteristics, clinical figures, and survival time among patients. This will assist clinicians in the treatment of HFM patients. We established that MCAO was mainly caused by lung cancer (53/98, 54.08%), esophageal cancer (22/98, 22.45%), and thyroid cancer (3/98, 3.06%). The median survival time of participants was 5.5 months. The survival rate was related to the primary disease, ECOG PS score, stent site, Hb, ALB, and serum LDH. Compared with the site of stent placement, the ECOG PS score is the primary factor in the survival rate of MCAO patients after airway stenting. However, clinicians should be cautious when applying the results of this study in clinical practice and should consider the medical needs of individual patients.

The article "Clinical Study of Airway Stent Implantation in the Treatment of Patients with Malignant Central Airway Obstruction" was published in 2022. Journal: Evid Based Complement Alternat Med.

## Figures and Tables

**Figure 1:** Kaplan-Meier curve showed the overall trend of survival rate with time.

**Figure 2:** Overall survival curve estimated using Kaplan-Meier. Comparison of survival rates based on (a) primary disease (*P*=0.044), (b) ECOG PS score (*P*=0.021), (c) stent placement site (*P* < 0.001), (d) LDH (*P*=0.082), (e) Hb (*P*=0.007), and (f) ALB (*P* < 0.001).

**Table 1:** Features of first airway stent placement in 98 MCAO patients.

Variable	Total number of cases (*n* = 98)
Anesthesia	—
Partial	72 (73.47%)
Anesthesia	26 (26.53%)
Stent	‒
Trachea	46 (46.94%)
Left main bronchus	19 (19.39%)
Right main bronchus	21 (21.43%)
Right middle bronchus	4 (4.08%)
Left main bronchus + right main bronchus	3 (3.06%)
Right middle bronchus + right distal bronchus	1 (1.02%)

**Table 2:** Log-rank analysis results of 98 MCAO patients after stent placement.

Feature	*n*	(95% CI) (month)	*P* value
Gender	—	—	0.562
Male	74	9.97 (6.68–13.25)	—
Female	24	13.79 (6.24–21.33)	—
Age	—	—	0.809
>60 years old	72	11.59 (7.72–15.46)	—
≤60 years old	26	9.09 (4.64–13.55)	—
With hypertension	—	—	0.685
No	52	9.67 (5.53–13.81)	—
Yes	46	12.00 (7.49–16.51)	—
With diabetes	—	—	0.632
No	87	11.38 (7.98–14.78)	—
Yes	11	8.09 (1.48–14.70)	—
Primary disease	—	—	0.044
Lung cancer	53	8.28 (5.12–11.44)	—
Esophageal cancer	22	11.33 (4.24–18.43)	—
Other∗	23	20.58 (9.64–31.53)	—
ECOG PS score	—	—	0.021
0–2 points	80	12.35 (8.83–15.86)	—
3–4 points	18	3.85 (0.96–6.73)	—
Treatment after stent placement	—	—	0.371
No treatment	22	11.82 (3.09–20.55)	—
Chemotherapy	21	8.51 (4.01–13.00)	—
Radiotherapy	14	15.33 (3.58–27.09)	—
Chemotherapy	31	11.61 (6.57–16.64)	—
Only receive supportive care	7	5.00 (0.35–9.66)	—
Stent	—	—	<0.001
Trachea	46	15.23 (9.94–20.51)	—
Left main bronchus	19	4.95 (2.13–7.77)	—
Right main bronchus	21	8.63 (5.34–11.91)	—
Other^†^	8	1.25 (0.45–2.05)	—
Hb (g/L)	—	—	0.007
<110	34	5.48 (3.24–7.72)	—
≥110	64	14.16 (9.37–18.94)	—
ALB (g/L)	—	—	<0.001
<40	60	6.64 (4.53–8.75)	—
≥40	38	23.22 (13.25–33.20)	—
Feature	n	(95% CI) (month)	*P* value
LDH (µg/L)	—	—	0.082
<250	68	12.21 (8.39–16.40)	—
≥250	30	5.51 (1.97–12.99)	—

∗Other diseases included airway stenosis, esophagotracheal fistula, lung infection, thyroid cancer, laryngeal cancer, tracheal space occupying, bronchial adenoid cystic carcinoma, mantle cell lymphoma. ^†^Other diseases included right middle bronchus, left main bronchus + right main Bronchus, and right middle bronchus + right distal bronchi. Hb: hemoglobin; ALB: albumin; LDH: serum lactate dehydrogenase.

**Table 3:** Survival factors and assignments of MCAO patients after airway stent placement.

Survival factors	Assignment
Gender	Female = 0, male = 1
Age	≤60 years old = 0, >60 years old = 1
Hypertension	No = 0, yes = 1
Diabetes	No = 0, yes = 1
Primary disease	Other∗ = 0, Lung cancer = 1, esophageal cancer = 2
ECOG PS score	0–2 points = 0, 3–4 points = 1
Treatment after stent placement	Radiotherapy = 0, chemotherapy = 1, Radiotherapy and chemotherapy = 2, Supportive Treatment = 3, No Treatment = 4
Stent	Trachea = 0, left main bronchus = 1, right main bronchus = 2, other^†^ = 3
Hb (g/L)	≥110 = 0, <110 = 1
ALB (g/L)	≥40 = 0, <40 = 1
LDH (µg/L)	<250 = 0, ≥250 = 1

∗Other diseases included airway stenosis, esophagotracheal fistula, lung infection, thyroid cancer, laryngeal cancer, tracheal space occupying, bronchial adenoid cystic carcinoma, and mantle cell lymphoma. ^†^Other diseases included right middle bronchus, left main bronchus + right main bronchus, and right middle bronchus + right distal bronchus. Hb: hemoglobin; ALB: albumin; LDH: serum lactate dehydrogenase.

The article "Clinical Study of Airway Stent Implantation in the Treatment of Patients with Malignant Central Airway Obstruction" was published in 2022. Journal: Evid Based Complement Alternat Med.

**Table 4:** Cox regression analysis results of 98 MCAO patients after stenting.

Factor	B	Se	Wald	*P* value	OR	95%CI
ECOG PS score	1.243	0.453	7.523	0.006	3.468	1.426–8.432
Stent	0.434	0.193	5.041	0.025	1.544	1.057–2.255

## Data Availability

The labeled dataset used to support the findings of this study are available from the corresponding author upon request.
